RETRACTED

# A Retrospective Study of Effectiveness of Thoracoscopic Lobectomy and Segmentectomy in Patients with Early-Stage Non-Small-Cell Lung Cancer

**DOI:** 10.1155/2022/6975236

**Published:** 2022-04-28

**Authors:** Jianning Xu, Lirong Huang, Yao Wang, Dongdong Guo, Jian Sun

**Affiliations:** Department of Cardiothoracic Surgery, Yancheng First Hospital, Affiliated Hospital of Nanjing University Medical School, Yancheng 224000, China

## Abstract

**Background:**

Surgical treatment is the first choice for non-small-cell lung cancer. To date, there are only few studies on the changes in laboratory indexes in two types of surgery, namely, thoracoscopic lobectomy and segmental pneumonectomy.

**Aim:**

To investigate the clinical impact of thoracoscopic lobectomy and segmentectomy in patients with early-stage non-small-cell lung cancer.

**Methods:**

We retrospectively reviewed the medical records of 94 patients with early-stage NSCLC in our hospital from October 2017 to October 2019. The patients were divided into two groups. The patients in control and observation groups received thoracoscopic lobectomy and thoracoscopic segmentectomy, respectively. The perioperative indicators, complications, lung function, T cell subsets, tumor markers, follow-up of tumor recurrence rate, and survival rate were compared between two groups.

**Results:**

The operation time of the observation group was longer, and the chest drainage volume was less at 24-48 h after the operation, and the chest tube indwelling time and postoperative hospital stay were shorter than those of the control group. No significant differences in complication probability were observed between two groups. The levels of FEV1, FVC, and MVV in the two groups were lower than those before the operation at 3 days after surgery, but the FEV1, FVC, and MVV levels in the observation group were higher than those in the control group. The CD3+, CD4+, and CD4+/CD8+ levels in the two groups were lower than those before the operation at 24 h and 72 h after the operation, but CD3+, CD4+, and CD4+/CD8+ levels in the observation group were higher than those of the control group.

**Conclusion:**

Thoracoscopic lobectomy and segmental resection have similar clinical effects in the treatment of early-stage NSCLC patients, but segmental resection can preserve healthy lung tissue as much as possible, with less trauma, protect lung function, and promote postoperative recovery.

## 1. Introduction

Lung cancer is the malignancy with the highest morbidity and mortality worldwide. Non-small-cell lung cancer (NSCLC) accounts for greater than 85% of all lung cancers [1]. For early-stage NSCLC, surgery remains the treatment of choice. Video-assisted thoracic surgery has the advantages of less trauma, less pain, and faster recovery for patients and has been widely developed in clinical practice [2]. Lobectomy and lymph node dissection are recognized as the standard treatment for early-stage NSCLC. However, resection of more lung tissue may affect postoperative quality of life [3]. Thoracoscopic segmentectomy can protect the lung tissue to the greatest extent and reduce surgical trauma, which has gradually attracted the attention of clinicians [4, 5]. At present, comparative studies on the two types of surgery mostly focus on the perioperative indexes and changes in lung function, and there are only few studies on the changes in laboratory indexes.

RETRACTED

We conducted a preliminary retrospective study using perioperative indicators, pulmonary function indexes (forced vital capacity in 1 s, forced vital capacity, and maximal voluntary ventilation), immune function (CD3+, CD4+, and CD4+/CD8+ levels), and tumor marker levels (cancer embryonic antigen, carbohydrate antigen 50, and cytokeratin 19 fragment) to compare the efficacy of thoracoscopic lobectomy and segmentectomy for early-stage NSCLC.

## 2. Materials and Methods

### 2.1. General Information

In this retrospective study, we included 94 patients with early-stage NSCLC in our hospital from October 2017 to October 2019. The patients were divided into two groups according to the surgery plan, with 47 patients in each group. Baseline information of the two groups was comparable (*P* > 0.05), as shown in Table 1.

### 2.2. Inclusion and Exclusion Criteria

#### 2.2.1. Inclusion Criteria

The inclusion criteria were as follows: (1) diagnosis of early-stage NSCLC histologically or cytologically; (2) absence of intrapulmonary or distant metastasis; (3) severe insufficiency of centroid, liver, kidney, and lung function; and (4) obtained informed consent from patients and their families.

#### 2.2.2. Exclusion Criteria

The exclusion criteria were as follows: (1) preoperative chemotherapy accompanied by radiotherapy, (2) no conversion to thoracotomy, (3) other malignant tumors, and (4) absence of chest surgery and severe chest trauma.

### 2.3. Methods

All patients were treated with double-lumen tracheal intubation under general anesthesia. The contralateral lung was ventilated and operated by the three-hole method. For the viewing aperture, a 1.0–1.5 cm incision was made in the seventh or eighth intercostal area of the midaxillary line. For the second aperture, a 1.0–2.0 cm incision was made in the seventh or eighth intercostal area at the posterior axillary line. For the main aperture, a 2.0–3.5 cm incision was made between the front axillary line and the midclavicular line in the fourth or fifth intercostal area. The intrapulmonary nodules were located. The control group underwent thoracoscopic lobectomy. The location of the lesion was explored to further define the lesion site, and the hilar tissue was dissected. The arteries, veins, and bronchus of the corresponding pulmonary lobes were dissected, and the pulmonary lobes to be resected were treated (cutting stapler). Lymph nodes were dissected, and a drainage tube was placed. The observation group underwent thoracoscopic pulmonary segmentectomy. The location of the lesion was explored, and the corresponding lung segments were dissected to fully expose the arteries, veins, and bronchus in the pulmonary segments. Arteries, veins, and segmental bronchus were treated. The segmental bronchus was clipped in front of the segmental bronchus, the lung was bulged, the boundary of the resected lung segment was confirmed, and the cutting suture device was used for treatment. Partial lung tissue adjacent to the lung segment can be resected to ensure adequate resection range. Bleeding was stopped completely, a drainage tube was placed, and sternal closure was performed.

RETRACTED

### 2.4. Observation Targets

Observation targets, including (1) perioperative indexes; (2) complications; (3) pulmonary function indexes (forced vital capacity in 1 s (FEV1), forced vital capacity (FVC), and maximal voluntary ventilation (MVV)), which were measured using the JAEGER MS Diffusion pulmonary function instrument (Jaeger AG, Germany), before and 3 days after surgery; (4) level of T cell subsets (CD3+, CD4+, and CD4+/CD8+) before surgery, 1 day after surgery, and 3 days after surgery (fasting venous blood (4 mL) was collected and centrifuged, and the T cell subsets were detected by FACSAria flow cytometry) (BD Company, USA); (5) serum tumor marker levels postoperation, 1 day, and 3 days after surgery (cancer embryonic antigen (CEA), carbohydrate antigen 50 (CA50), and cytokeratin 19 fragment (CYFRA21-1)) (CEA and CA50 were detected by radioimmunoassay, and CYFRA21-1 was detected by electrochemical process); and (6) tumor recurrence and survival rates of the two groups, were analyzed after 2 years of follow-up.

### 2.5. Statistical Analysis

The Statistical Package for the Social Sciences, version 22.0, software program was used for statistical analysis. Numbers are expressed as rates. *χ*^2^ test was used for comparison between the two groups. Measurement data conforming to normal distribution are represented as ($\bar{\text{x}}\pm \text{s}$), and the independent sample t*-*test was used for comparison between the groups. *P* < 0.05 was considered to indicate statistical significance.

RETRACTED

## 3. Results

### 3.1. Perioperative Indicators

There was no significant difference in the amount of intraoperative blood loss and the number of lymph nodes resected between the observation group (168.29 ± 69.75 mL and 11.85 ± 2.57 mL) and the control group (179.37 ± 74.28 mL and 12.56 ± 2.63 mL) (*P* > 0.05). The operation time of the observation group (170.41 ± 14.82 min) was longer than that of the control group (150.29 ± 17.05 min), the thoracic drainage volume within 24–48 h after the operation was lower in the observation group (139.26 ± 42.82 mL) than in the control group (172.54 ± 45.16 mL), and the chest tube duration and postoperative time of the observation group (4.05 ± 0.71 d and 6.74 ± 1.25 d) were shorter than those of the control group (4.81 ± 0.83 d and 8.16 ± 1.37 d) (*P* < 0.05), as shown in Table 2.

### 3.2. Complications

There was no significant difference in complication probability between the observation group (6.38%) and the control group (10.64%) (*P* > 0.05), as shown in Table 3.

### 3.3. Pulmonary Function Index

There were no significant differences in FEV1, FVC, and MVV levels between the observation group (2.48 ± 0.50, 2.86 ± 0.57, and 78.65 ± 9.94 L, respectively) and the control group (2.53 ± 0.54, 2.92 ± 0.54, and 80.02 ± 10.26 L, respectively) before surgery (*P* > 0.05). Three months after operation, FEV1, FVC, and MVV levels in both groups were lower than those before the operation. However, FEV1, FVC, and MVV levels in the observation group (2.04 ± 0.49, 2.39 ± 0.47, and 69.35 ± 7.26 L, respectively) were higher than those in the control group (1.65 ± 0.43, 1.98 ± 0.45, and 58.47 ± 6.84 L, respectively) (*P* < 0.05), as shown in Table 4.

### 3.4. T Cell Subsets

There were no significant differences of the levels of CD3+, CD4+, and CD4+/CD8+ between the observation group (66.23 ± 4.94%, 36.71 ± 4.48%, and 1.53 ± 0.19%, respectively) and the control group (65.31 ± 5.42%, 35.92 ± 5.01%, and 1.49 ± 0.22%, respectively) before the operation (*P* > 0.05). The levels of CD3+, CD4+, and CD4+/CD8+ in both groups at 24 and 72 h after surgery were lower than those before the surgery, but the levels of CD3+ and CD4+/CD8+ (CD3+ [57.51 ± 5.11% and 62.08 ± 5.32%], CD4+ [30.05 ± 4.09% and 33.20 ± 4.26%], and CD4+/CD8+ [1.29 ± 0.17% and 1.41 ± 0.18%]) were higher in the observation group than in the control group (CD3+ [51.28 ± 4.83% and 57.53 ± 5.16%], CD4+ [25.37 ± 3.95% and 28.93 ± 5.07%], and CD4+/CD8+ [1.14 ± 0.18% and 1.24 ± 0.19%]) (*P* < 0.05), as shown in Table 5.

### 3.5. Tumor Marker

There were no significant differences in the levels of serum CEA, CA50, and CYFRA21-1 between the observation group (21.29 ± 5.92 ng/mL, 25.36 ± 5.47 U/mL, and 5.19 ± 0.57 ng/mL, respectively) and the control group (22.37 ± 4.61 ng/mL, 26.07 ± 6.05 U/mL, and 5.03 ± 0.64 ng/mL, respectively) before surgery (*P* > 0.05). The levels of serum CEA, CA50, and CYFRA21-1 in the observation group at 24 and 72 h after surgery were lower than those before surgery. CEA, CA50, and CYFRA21-1 Levels in the observation group (CEA [9.95 ± 2.09 and 8.04 ± 1.58 ng/mL], CA50 [10.49 ± 2.46 and 8.53 ± 1.69 U/mL], and CYFRA21-1 [2.48 ± 0.39 and 1.97 ± 0.38 ng/mL]) were lower than those in the control group (CEA [12.03 ± 2.21 and 9.87 ± 1.86 ng/mL], CA50 [12.55 ± 2.67 and 10.08 ± 1.72 U/mL], and CYFRA21-1 [3.10 ± 0.51 and 2.53 ± 0.44 ng/mL]) (*P* <0.05), as shown in Table 6.

RETRACTED

### 3.6. Cancer Recurrence and Survival Rates

Both groups were followed up for 2 years. Two patients in the observation group and three patients in the control group were lost to follow-up. There was no tumor-related death during follow-up in either group. Local recurrence was observed in 2 (4.44%) patients in the observation group and 1 (2.27%) patient in the control group. There was no significant difference in the local recurrence rate between the two groups (*χ*^2^ = 0.32, *P* = 0.570).

## 4. Discussion

Currently, NSCLC is primarily treated with minimally invasive procedures, including video-assisted thoracoscopic surgery and smaller resection of the primary lesion [6, 7]. Lobectomy and lymph node dissection are the standard treatment approaches for early-stage NSCLC. However, this finding is not consistent with the minimally invasive concept of achieving better outcomes with less trauma [8]. In recent years, segmentectomy has been used to treat early-stage NSCLC. Studies have shown that there are no significant differences between thoracoscopic segmentectomy and lobectomy in the number of lymph nodes resected, postoperative complications, and local recurrence rates. However, segmentectomy has the advantages of less trauma, quick recovery, and protection of lung function [9, 10].

Operation duration is one of the important indexes to evaluate the operative method. In this study, the operation time of the observation group was longer than that of the control group (*P* < 0.05), which was consistent with the result of a previous study [11]. Considering that this study was related to more complex clinical anatomy of pulmonary segments, it may also be caused by unskilled operation and the existence of a learning curve. In this study, the thoracic drainage volume 24–48 h after surgery between the two groups was compared. The thoracic drainage volume 24–48 h after surgery was easily affected by intraoperative residual rinse fluid, and the chest tube indwelling time was significantly affected by the third 24 h. Therefore, the thoracic drainage volume 24–48 h after surgery could better reflect the effect of trauma on the drainage volume change. The observation group had lower thoracic drainage volume 24–48 h after surgery than the control group, and the durations of chest tube indwelling and postoperative hospitalization were shorter in the observation group than in the control group (*P* < 0.05). This indicates that thoracoscopic segmentectomy resection can reduce surgical trauma to a certain extent and promote postoperative recovery of patients. Lymphadenectomy is an important indicator for radical resection of lung cancer. In this study, there was no significant difference in the number of lymph nodes resected between the two groups, indicating that the effectiveness of thoracoscopic segmentectomy was similar to that of lobotomy (*P* > 0.05), which was consistent with the results of previous studies [12, 13]. In addition, there was no significant difference in the incidence of complications between the two groups (*P* > 0.05), indicating similar safety between the two procedures.

RETRACTED

The National Comprehensive Cancer Network suggests segmentectomy for patients with poor pulmonary reserve, for which lobectomy is not possible. A number of studies have shown that segmentectomy in patients with early-stage NSCLC can better protect lung function after surgery, which is of great significance for patients with basic pulmonary diseases, such as chronic bronchitis and emphysema, or elderly patients with poor lung function [14–16]. Data from this study showed that 3 days after surgery, the FEV1, FVC, and MVV levels in both groups were lower than those before surgery, but these levels in the observation group were higher than those in the control group (*P* < 0.05), indicating the advantages of thoracoscopic pulmonary segmentectomy to protect lung function. The reasons for this finding are as follows: (1) Segmentectomy can preserve healthy lung tissue to the maximum extent and has a direct protective effect on lung function, and (2) after lobectomy, the remaining lobes dilated, the angle of bronchus changed, the original shape of the bronchus changed, the airway narrowed, and the airway resistance increased. However, segmentectomy can protect lung function to a certain extent because of small dilatation and small change of bronchial angle [17].

Immunosuppression is a common complication of surgery, and surgical trauma and stress reaction are closely related to its occurrence [18, 19]. Immunosuppression can lead to nosocomial infection and tumor spread. Therefore, it is of great significance to understand the effect of surgical trauma on the immune function of patients with NSCLC. The antitumor immunological effect of the body is mainly cellular immunity, and T cells are the main effector cells of cellular immunity. Data in this study showed that levels of CD3+, CD4+, and CD4+/CD8+ in the two groups 24 and 72 h after surgery were lower than those before surgery, but those in the observation group were higher than those in the control group (*P* < 0.05), indicating less immunosuppression caused by thoracoscopic segmentectomy and the advantages of segmentectomy. CEA, CA50, and CYFRA21-1 are all typical tumor markers of lung cancer [20]. In this study, the levels of serum CEA, CA50, and CYFRA21-1 in both groups significantly decreased 24 h and 72 h after surgery, which was considered to be related to the reduction of postoperative tumor load. However, the levels of serum CEA, CA50, and CYFRA21-1 in the observation group were lower than those in the control group 24 h and 72 h after surgery. The reasons may be that segmentectomy has less trauma and less stress response, which can reduce the degree of blood cancer metastasis induced by trauma inflammation. However, the exact mechanism remains to be further discussed.

RETRACTED

However, this study had a limitation. This was a single-center and small-sample study; therefore, whether the results of the study are broadly effective still needs to be confirmed by further clinical investigations.

## 5. Conclusion

In conclusion, the clinical efficacy of thoracoscopic lobectomy and segmentectomy for patients with early-stage NSCLC is similar. However, segmentectomy can maximize the preservation of healthy lung tissue with less trauma, protect lung function, promote postoperative recovery, and reduce the effect of stress response on immune function and serum tumor marker levels.

## Figures and Tables

**Table 1:** Comparison of baseline data between the two groups.

Information	Control group (*n* = 47)	Observation group (*n* = 47)	t/*χ*^2^	*P*
Gender (male/female)	28/19	30/17	0.180	0.671
Age	36~77 (58.09 ± 7.73)	35~78 (59.14 ± 8.25)	0.637	0.526
BMI (kg/m^2^)	17~28 (22.91 ± 1.76)	17~28 (23.11 ± 2.08)	0.503	0.616
Tumor diameter (cm)	0.5~2.0 (1.68 ± 0.15)	0.5~2.0 (1.64 ± 0.16)	1.250	0.214
TNM staging				
0 stage	2 (4.26)	1 (2.13)	0.474	0.789
IA stage	39 (82.98)	41 (87.23)		
IB stage	6 (12.77)	5 (10.64)		
Pathology				
Adenocarcinoma	36 (76.60)	38 (80.85)	0.446	0.800
Squamous carcinoma	9 (19.15)	8 (17.02)		
Others	2 (4.26)	1 (2.13)		
Complications				
Hypertension	3 (6.38)	1 (2.13)	1.044	0.307
Diabetes	2 (4.26)	1 (2.13)	0.001	1.000
Coronary heart disease	1 (2.13)	2 (4.26)	0.001	1.000

BMI: body mass index; TNM: tumor, nodes, and metastases.

RETRACTED

**Table 2:** Comparison of perioperative indicators between the two groups ($\bar{x}\pm s$).

Indicators	Observation group (*n* = 47)	Control group (*n* = 47)	t	*P*
Intraoperative blood loss (mL)	168.29 ± 69.75	179.37 ± 74.28	0.745	0.458
Operation time (min)	170.41 ± 14.82	150.29 ± 17.05	6.106	0.001
Number of lymph nodes removed	11.85 ± 2.57	12.56 ± 2.63	1.324	0.189
24-48 h postoperative thoracic drainage volume (mL)	139.26 ± 42.82	172.54 ± 45.16	3.666	0.001
Chest tube duration (d)	4.05 ± 0.71	4.81 ± 0.83	4.770	0.001
Hospital stays (d)	6.74 ± 1.25	8.16 ± 1.37	5.249	0.001

**Table 3:** Comparison of complications between the two groups (*n* %).

Groups	Number of cases	Pulmonary air leakage	Lung infection	Incision infection	Chylothorax	Total incidence
Observation group	47	1 (2.13)	1 (2.13)	1 (2.13)	0 (0.00)	3 (6.38)
Control group	47	1 (2.13)	2 (4.26)	1 (2.13)	1 (2.13)	5 (10.64)
*χ* ^2^						0.547
*P*						0.460

**Table 4:** Comparison of pulmonary function indexes between the two groups ($\bar{x}\pm s$, L).

Groups	Number of cases	FEV1		FVC		MVV	
		Presurgery	3 months after surgery	Presurgery	3 months after surgery	Presurgery	3 months after surgery
Observation group	47	2.48 ± 0.50	2.04 ± 0.49^a^	2.86 ± 0.57	2.39 ± 0.47^a^	78.65 ± 9.94	69.35 ± 7.26^a^
Control group	47	2.53 ± 0.54	1.65 ± 0.43^a^	2.92 ± 0.54	1.98 ± 0.45^a^	80.02 ± 10.26	58.47 ± 6.84^a^
*t*		0.466	4.101	0.524	4.320	0.657	7.478
*P*		0.643	0.001	0.602	0.001	0.513	0.001

Note: ^a^*P* < 0.05, compared with the group before surgery. FEV1: forced vital capacity in 1 second; FVC: forced vital capacity; MVV: maximal voluntary ventilation.

**Table 5:** Comparison of T cell subsets between the two groups ($\bar{x}\pm s$).

Groups	Number of cases	CD3^+^ (%)			CD4^+^ (%)			CD4^+^/CD8^+^		
		Presurgery	24 h after surgery	72 h after surgery	Presurgery	24 h after surgery	72 h after surgery	Presurgery	24 h after surgery	72 h after surgery
Observation group	47	66.23 ± 4.94	57.51 ± 5.11^a^	62.08 ± 5.32^a^	36.71 ± 4.48	30.05 ± 4.09^a^	33.20 ± 4.26^a^	1.53 ± 0.19	1.29 ± 0.17^a^	1.41 ± 0.18^a^
Control group	47	65.31 ± 5.42	51.28 ± 4.83^a^	57.53 ± 5.16^a^	35.92 ± 5.01	25.37 ± 3.95^a^	28.93 ± 5.07^a^	1.49 ± 0.22	1.14 ± 0.18^a^	1.24 ± 0.19^a^
*t*		0.860	6.074	4.209	0.806	5.643	4.421	0.943	4.153	4.453
*P*		0.392	0.001	0.001	0.422	0.001	0.001	0.348	0.001	0.001

Note: ^a^*P* < 0.05, compared with the group before surgery.

**Table 6:** Comparison of serum tumor marker levels between the two groups ($\bar{x}\pm s$).

Groups	Number of cases	CEA (ng/mL)			CA50 (U/mL)			CYFRA21-1 (ng/mL)		
		Presurgery	24 h after surgery	72 h after surgery	Presurgery	24 h after surgery	72 h after surgery	Presurgery	24 h after surgery	72 h after surgery
Observation group	47	21.29 ± 5.92	9.95 ± 2.09^a^	8.04 ± 1.58^a^	25.36 ± 5.47	10.49 ± 2.46^a^	8.53 ± 1.69^a^	5.19 ± 0.57	2.48 ± 0.39^a^	1.97 ± 0.38^a^
Control group	47	22.37 ± 4.61	12.03 ± 2.21^a^	9.87 ± 1.86^a^	26.07 ± 6.05	12.55 ± 2.67^a^	10.08 ± 1.72^a^	5.03 ± 0.64	3.10 ± 0.51^a^	2.53 ± 0.44^a^
*t*		0.987	4.688	5.141	0.597	3.890	4.407	1.280	6.620	6.604
*P*		0.326	0.001	0.001	0.552	0.001	0.001	0.204	0.001	0.001

Note: ^a^*P* < 0.05, compared with the group before surgery. CEA: cancer embryonic antigen; CA: carbohydrate antigen; CYFRA: cytokeratin 19 fragment.

RETRACTED

## Data Availability

The authors confirm that the data supporting the findings of this study are available within the article.

## References

[1] Wu F., Zhou H., Li F., Wang J. T., Ai T. (2018). Spectral CT imaging of lung cancer: quantitative analysis of spectral parameters and their correlation with tumor characteristics. *Academic Radiology*.

[2] Mimae T., Okada M. (2020). Are segmentectomy and lobectomy comparable in terms of curative intent for early stage non-small cell lung cancer?. *General Thoracic and Cardiovascular Surgery*.

[3] Aokage K., Yoshida J., Hishida T. (2017). Limited resection for early-stage non-small cell lung cancer as function-preserving radical surgery: a review. *Japanese journal of clinical oncology*.

[4] Jones G. D., Caso R., Choe G. (2021). Intentional segmentectomy for clinical T1 N0 non-small cell lung cancer: survival differs by segment. *The Annals of Thoracic Surgery*.

[5] Stamatis G., Leschber G., Schwarz B. (2019). Perioperative course and quality of life in a prospective randomized multicenter phase III trial, comparing standard lobectomy *vs* anatomical segmentectomy in patients with non-small cell lung cancer up to 2 cm, stage IA (7th edition of TNM staging system). *Lung Cancer*.

[6] Tan C. L., Lim T. H., Lim T. K. (2016). Concordance of anaplastic lymphoma kinase (ALK) gene rearrangements between circulating tumor cells and tumor in non-small cell lung cancer. *Oncotarget*.

[7] Suzuki K., Saji H., Aokage K. (2019). Comparison of pulmonary segmentectomy and lobectomy: safety results of a randomized trial. *The Journal Of Thoracic And Cardiovascular Surgery*.

[8] Voltolini L., Gonfiotti A., Viggiano D., Borgianni S., Farronato A., Bongiolatti S. (2020). Extended sleeve-lobectomy for centrally located locally advanced non-small cell lung cancer is a feasible approach to avoid pneumonectomy. *Journal of Thoracic Disease*.

[9] Hong T. H., Cho J. H., Shin S. (2018). Extended sleeve lobectomy for centrally located non-small-cell lung cancer: a 20-year single-centre experience. *European Journal of Cardio-Thoracic Surgery*.

RETRACTED

[10] Olland A., Falcoz P. E. (2020). Complex segmentectomy in the treatment of stage IA non-small-cell lung cancer. *European Journal of Cardio-Thoracic Surgery*.

[11] Deng H. Y., Tang X. (2020). Is less more for early-stage non-small-cell lung cancer? Current evidence for performing segmentectomy. *European Journal of Cardio-Thoracic Surgery*.

[12] Widder J., Van De Wauwer C., Langendijk J. A. (2017). Lobectomy or sublobectomy for small non-small-cell lung cancer: the question remains. *Journal of Clinical Oncology*.

[13] Seguin-Givelet A., Lutz J., Brian E., Grigoroiu M., Gossot D. (2018). Surgical treatment of early stage non-small cell lung cancer by thoracoscopic segmental resection. *Revue Des Maladies Respiratoires*.

[14] Dolan D. P., White A., Mazzola E. (2021). Outcomes of superior segmentectomy versus lower lobectomy for superior segment stage I non-small-cell lung cancer are equivalent: an analysis of 196 patients at a single, high volume institution. *Journal of Surgical Oncology*.

[15] Smith S. P., Bograd A. J., Levy G. (2021). Surgical management of non-small cell lung cancer invading the fissure: less is more?. *The Annals Of Thoracic Surgery*.

[16] Deng Y., Wang J., Mu J., Wang Z., Wang G. (2020). Complete uniportal thoracoscopic anatomic lung resection with systematic mediastinal lymphadenectomy for non-small cell lung cancer: personal experience of 326 cases. *Surgical Laparoscopy, Endoscopy & Percutaneous Techniques*.

[17] Zhang Y., Gao Y. (2016). Effects of VATS lobectomy, VATS anatomic segmentectomy, and open thoracotomy on pulmonary function of patients with non-small cell lung cancer. *Zhongguo Fei Ai Za Zhi*.

[18] De Bari B., Durham A., Bourhis J., Ozsahin M. (2017). Can segmentectomy still be proposed as an alternative to lobectomy in 2016?. *Journal of Clinical Oncology: Official Journal of the American Society of Clinical Oncology*.

[19] Amore D., Casazza D., Bergaminelli C. (2019). Left lower lobectomy and partial preservation of segmental arteries of left upper lobe: a strategy to avoid pneumonectomy in selected cases. *Thoracic Cancer*.

[20] Pennell N. A., Arcila M. E., Gandara D. R., West H. (2019). Biomarker testing for patients with advanced non-small cell lung cancer: real-world issues and tough choices. *American Society of Clinical Oncology Educational Book*.

